RETRACTED

# +HOXA10-AS Promotes Malignant Phenotypes of Gastric Cancer via Upregulating HOXA10

**DOI:** 10.1155/2022/1846687

**Published:** 2022-02-16

**Authors:** Fengyu Cao, Yongbin Zheng, Chao Yang, Suoyang Huang, Xiaobo He, Shilun Tong

**Affiliations:** Department of Gastrointestinal Surgery, Renmin Hospital of Wuhan University, Wuhan, Hubei 430060, China

## Abstract

**Objective:**

To study the role of long noncoding RNA HOXA10-AS in gastric cancer (GC) and its underlying mechanism which is one of the most common and fetal malignancies. Long noncoding RNA HOXA10-AS is highly expressed and acts in an oncogenic role in cancers. However, its roles in GC are still unknown.

**Methods:**

The expression of HOXA10-AS and HOXA10 in GC tissues from the TCGA database was analyzed. Western blot and qRT-PCR assays were applied to examine the expression of HOXA10-AS and HOXA10. Cell proliferation was evaluated with CCK-8 and EdU incorporation assays. Cell apoptosis was analyzed by flow cytometry. Migratory and invasive capacities were evaluated with wound healing and transwell assays.

**Results:**

HOXA10-AS and HOXA10 were upregulated in GC, and their expressions were positively correlated. Knockdown of HOXA10-AS inhibited HOXA10 expression in GC cells. Furthermore, knockdown of HOXA10-AS restrained GC cell proliferation, migration, and invasion but promoted apoptosis. In addition, overexpression of HOXA10-AS promoted malignant phenotypes of GC cells, but all these effects could be reversed by knockdown of HOXA10.

**Conclusion:**

HOXA10-AS promoted GC cell proliferation, migration and invasion and enhanced apoptosis via upregulating HOXA10. Our study implies a novel regulatory mechanism of malignant phenotypes and provides potential therapeutic targets for GC.

## 1. Introduction

GC generally occurs in the inner lining of the stomach and is one of the most common and fatal malignancies [1], causing 769,000 deaths in 2020 [2]. Surgical resection with adjuvant chemoradiation or chemotherapy is the major treatment for GC [3, 4]. Despite growing advances have been made in surgical approaches, immunotherapy, and molecular-targeted therapy in recent years [3, 5], the improvement of survival of GC patients is not intriguing, especially for advanced patients. GC diagnosed at a distant stage shows poor prognosis and a low five-year survival rate of 5.3% [6]. Thus, it is essential to elucidate the pathogenesis of GC and seek key regulators in GC for developing novel therapeutic strategies.

Long noncoding RNAs (lncRNAs) have attracted much attention because of their key roles in the regulation of various cancers [7]. lncRNAs have oncogenic or antitumor activities and exert important roles in the onset and progression of cancers, which offers potential therapeutic opportunities [8, 9]. For instance, lncRNA CAR10 was upregulated in lung adenocarcinoma, and lncRNA CAR10 enhanced metastasis via acting as a miRNA sponge and regulating SNAI expression [10]. Zou et al. found that lncRNA 00324 was upregulated in GC, and lncRNA 00324 enhanced GC cell proliferation, migration, and invasion and restrained apoptosis by binding to HuR and maintaining the stability of FAM83B [11].

RETRACTED

Several lncRNAs are implicated in GC, such as HOTAIR [12], NEAT1 [13], and LINC01410 [14]. HOXA10 antisense RNA (HOXA10-AS) is a lncRNA and transcribed antisense to HOXA10 [15]. Intriguingly, HOXA10-AS is upregulated and functions as an oncogene in various cancers including leukemia [15], glioma [16], and oral cancer [17]. Dong and colleagues reported that HOXA10-AS expression was elevated in glioma, and HOXA10-AS promoted glioma cell proliferation and enhanced apoptosis via activating HOXA10 expression [16]. However, the role of HOXA10-AS in GC remains a mystery.

HOXA10 belongs to the HOXA gene family and plays key roles in uterine embryogenesis and embryo implantation [18]. Importantly, HOXA10 is highly expressed in several cancers and exerts an oncogenic activity [19, 20]. Song et al. demonstrated that HOXA10 expression was increased in GC, and it suppressed apoptosis and promoted proliferation [21]. Moreover, Chen et al. reported that overexpression of HOXA10 facilitated cell proliferation and tumorigenesis and reduced apoptosis in GC via activating the JAK1/STAT3 signaling [22]. However, the interaction between HOXA10-AS and HOXA10 and its role in GC have not been elucidated.

In this study, we aimed to investigate whether HOXA10-AS regulates malignant phenotypes including proliferation, apoptosis, migration, and invasion of GC cells via modulating HOXA10 expression, which will deepen understanding of GC progression and provide potential therapeutic targets for GC.

## 2. Methods

### 2.1. Patients

All patients were informed and provided written consent, and our study was approved by the Ethics Committee of Renmin Hospital of Wuhan University. GC and adjacent normal (NC) tissues were obtained from 70 patients diagnosed with GC and snap-frozen in liquid nitrogen. Overall survival was monitored for 60 months. Clinical pathological characteristics were exhibited in Table 1.

### 2.2. Cell Culture and Transfection

Human gastric cancer cells HGC-27 and AGS and normal gastric mucosal epithelial cell GES-1 were obtained from the American Type Culture Collection (ATCC, Manassas, VA, USA). Cells were maintained in Roswell Park Memorial Institute (RPMI) 1640 (Sartorius, Göttingen, Germany) containing 10% fetal bovine serum (Solarbio, Beijing, China) at 37°C. Briefly, cells were grown to 80% confluency and detached using Trypsin-EDTA (0.25%, Thermo Fisher, Waltham, MA, USA) for subculture. Culture medium was replaced every 24 hours.

RETRACTED

HOXA10-AS was cloned into pcDNA3.1 (HOXA10-AS) for overexpression. siRNAs against HOXA10-AS (si-HOXA10-AS#1, #2, and #3) and HOXA10 (si-HOXA10) and negative controls (si-NC) were purchased from Ribobio (Guangzhou, China). Cells were transfected with si-NC, si-HOXA10-AS (#1, #2, and #3), empty vector, HOXA10-AS, or HOXA10-AS in combination with si-HOXA10 using Lipo3000 reagent (Thermo Fisher) following the manual. After 48-72 hours, cells were harvested for subsequent assays.

### 2.3. Real-Time Quantitative PCR (qRT-PCR)

Prior to RNA extraction, GC and NC tissues were snap-frozen in liquid nitrogen and homogenized. Total RNA was extracted from tissue homogenates and HGC-27, AGS, and GES-1 cells using TRIzol reagent (Thermo Fisher). Subsequently, RNA was reversely transcribed into cDNA, and real-time quantitative PCR was applied to analyze the expression of HOXA10-AS and HOXA10. GAPDH was used as a normalization control. The 2^−∆∆Ct^ method was used for calculation. Primers are listed in Supplementary Table 1.

### 2.4. Cell Counting Kit-8 (CCK-8) Assay

The CCK-8 assay was performed as previously described [23]. HGC-27 and AGS cells were seeded and incubated in 96-well plates for 0, 24, 48, or 72 hours. Media were replaced with 100 *μ*L of fresh media, and 10 *μ*L of CCK-8 (Dojindo, Kumamoto, Japan) was added. Cells were incubated for an additional 4 hours, and the absorbance at 450 nm was recorded.

### 2.5. Cell Apoptosis

Apoptosis was evaluated with Annexin V-FITC Apoptosis Detection Kit from Beyotime (Shanghai, China) as previously described [24]. In brief, 1 × 10^5^ cells were resuspended in a binding buffer (100 *μ*L) and stained with Annexin V-FITC and propidium iodide for 20 minutes. Apoptosis was examined using a CytoFLEX flow cytometer (Beckman Coulter, Indianapolis, IN, USA).

### 2.6. 5-Ethynyl-2'-Deoxyuridine (EdU) Incorporation

HGC-27 and AGS cells were seeded on coverslips and incubated in RPMI 1640 media supplemented with EdU (10 *μ*M) for 16 hours. Subsequently, cells were fixed using 4% formaldehyde in PBS for 15 minutes and permeabilized in 0.5% Triton X-100 solution. The EdU staining reaction cocktail was prepared as suggested in the manual and added into cells. After incubation for half an hour, cells were stained with DAPI (Beyotime) and mounted with antifade mounting medium for imaging.

### 2.7. Transwell Assay

Transwell assays were performed as previously described [25]. Upper chambers of Transwell inserts with 8.0 *μ*m pore provided by Corning (Corning, NY, USA) were precoated with Matrigel (BD, Franklin Lakes, NJ, USA). HGC-27 and AGS cells were seeded on the upper chambers and cultured for 24 hours. Cells invaded into the lower chambers, which were fixed and stained with 1% crystal violet solution (Sigma, St. Louis, MO, USA) for imaging under a microscope from Olympus.

RETRACTED

### 2.8. Wound Healing Assay

Wound healing assays were performed as previously described [25]. HGC-27 and AGS cells were plated and cultured into a confluent monolayer. Scratches were made on cell monolayers using cell combs from EMD Millipore (Darmstadt, Germany), and cells were cultured for wound healing. The wound healing was quantified using ImageJ software.

### 2.9. Western Blot

GC cells were lysed in radioimmunoprecipitation assay (RIPA) lysis buffer (Boster, Pleasanton, CA, USA), and supernatants were collected. Protein was quantified with a BCA kit (Abcam, Cambridge, UK). Protein (40 *μ*g) was electrophoresed and transferred to polyvinylidene fluoride (PVDF) membranes (GE, Waukesha, WI, USA). Membranes were blocked in 8% nonfat milk solution and incubated with a goat polyclonal antibody against HOXA10 (1 : 1000, Abcam) overnight. Next day, membranes were rinsed and incubated with a horseradish peroxidase- (HRP-) labeled secondary antibody. Enhanced chemiluminescence (ECL) substrates (Bio-Rad, Hercules, CA, USA) were used for visualizing bands. The ImageJ software was used to analyze band intensity.

### 2.10. Statistical Analysis

All assays were repeated at least three times, and data was shown as mean ± standard deviation. The Kaplan Meier curve was applied to analyze the survival of HOXA10-AS^high^ and HOXA10-AS^low^ patients. The correlation of HOXA10-AS and HOXA10 was analyzed using Spearman's correlation. The variance of two groups was analyzed with Student's *t* test. One-way analysis of variance (ANOVA) was used for comparing more than two groups. The GraphPad Prism 8.0 software (GraphPad Software, San Diego, CA, USA) was used to analyze the data. *p* < 0.05 was statistically significant. ^∗^*p* < 0.05, ^∗∗^*p* < 0.01, and ^∗∗∗^*p* < 0.001.

## 3. Results

### 3.1. HOXA10-AS Was Highly Expressed in GC Tissues and Cells

To explore the function of HOXA10-AS in GC, we analyzed HOXA10-AS expression using the TCGA database and found elevated HOXA10-AS expression in stomach adenocarcinoma (STAD, Figure 1(a)). Elevated expression of HOXA10-AS was also observed in GC tissues from patients (Figure 1(b)). According to the median expression level of HOXA10-AS, GC patients were divided into two groups, HOXA10-AS^high^ and HOXA10-AS^low^. HOXA10-AS^high^ patients showed obvious poor survival compared to HOXA10-AS^low^ patients (Figure 1(c)). The expression of HOXA10-AS was significantly correlated with lymph node metastasis; tumor, node, and metastasis (TNM) stage; and differentiation rather than age, gender, and tumor size (Table 1). In addition, we analyzed the HOXA10-AS expression in HGC27 and AGS GC cells and normal human gastric mucosal epithelial cell GES-1. As shown in Figure 1(d), GC cells showed a higher expression of HOXA10-AS than GES-1 cells. These observations suggested that HOXA10-AS was upregulated in GC, and its high expression indicated poor prognosis.

RETRACTED

### 3.2. Knockdown of HOXA10-AS Suppressed GC Cell Proliferation and Enhanced Apoptosis

To investigate whether HOXA10-AS regulates malignant phenotypes, HOXA10-AS was knocked down in HGC27 and AGS cells through transfection of siRNAs against HOXA10-AS (si-HOXA10-AS#1, #2, and #3, Figure 2(a)). Si-HOXA10-AS#1 exhibited highest knockdown efficiency (Figure 2(a)), and it was selected for subsequent knockdown assays (hereafter, referred to as si-HOXA10-AS). CCK-8 assays showed that knockdown of HOXA10-AS significantly inhibited cell proliferation (Figure 2(b)). Besides, knockdown of HOXA10-AS reduced EdU incorporation in HGC27 and AGS cells (Figure 2(c)). Furthermore, compared to si-NC, si-HOXA10-AS significantly enhanced GC cell apoptosis (Figure 2(d)). Collectively, these data demonstrated that knockdown of HOXA10-AS restrained GC cell proliferation and enhanced apoptosis.

### 3.3. Knockdown of HOXA10-AS Suppressed GC Cell Migration and Invasion

We further analyzed whether knockdown of HOXA10-AS affected GC cell migration and invasion by wound healing and transwell assays. We observed that the wound healing of HGC27 and AGS cells with knockdown of HOXA10-AS was slowed down, suggesting that knockdown of HOXA10-AS suppressed GC cell migration (Figure 3(a)). Furthermore, compared to control cells, HGC27 and AGS cells with knockdown of HOXA10-AS exhibited reduced invasive capacity (Figure 3(b)). Therefore, knockdown of HOXA10-AS impaired migratory and invasive capacities of GC cells.

### 3.4. HOXA10-AS Promoted HOXA10 Expression in GC Cells

We proposed that HOXA10-AS might regulate HOXA10 expression. By analyzing the TCGA database, we observed increased expression of HOXA10 in STAD (Figure 4(a)). The expression of HOXA10-AS and HOXA10 was positively correlated (Figure 4(b)). We also analyzed HOXA10 expression in GC and NC tissues from patients. Consistently, we observed elevated expression of HOXA10 in GC (Figure 4(c)). Furthermore, HOXA10-AS expression was positively correlated with HOXA10 expression (Figure 4(d)). Additionally, HOXA10 expression was obviously reduced by knockdown of HOXA10-AS in GC cells (Figure 4(e)). Taken together, these results demonstrated that HOXA10-AS promoted HOXA10 expression in GC.

RETRACTED

### 3.5. HOXA10-AS Accelerated Malignant Phenotypes of GC via Promoting HOXA10 Expression

To further explore whether HOXA10-AS-mediated regulation of GC is dependent on regulating HOXA10 expression, GC cells were transfected with HOXA10-AS-overexpressing vector in combination with siRNA against HOXA10 (si-HOXA10). HOXA10-AS was efficiently overexpressed in HGC27 and AGS cells (Figure 5(a)). HOXA10-AS overexpression-induced high expression of HOXA10 was inhibited by knockdown of HOXA10 in HGC27 and AGS cells (Figure 5(b)). CCK-8 and EdU incorporation assays showed that overexpression of HOXA10-AS facilitated cell proliferation, which was reversed by knockdown of HOXA10 (Figures 5(c) and 5(d)). Moreover, overexpression of HOXA10-AS-mediated inhibition of GC cell apoptosis was largely rescued by knockdown of HOXA10 (Figure 5(e)). Overexpression of HOXA10-AS contributed to GC cell migration and invasion, which were abrogated by knockdown of HOXA10 (Figures 5(f) and 5(g)). To conclude, HOXA10-AS promoted malignant phenotypes of GC cells via regulating HOXA10 expression.

## 4. Discussion

GC affects tens of millions of patients and causes serious health issues [26, 27]. In 2020, more than one million new patients are reported, and GC is responsible for 769,000 deaths, which makes GC the 5th most common malignancy and the 4th cause of cancer mortality [28]. The five-year survival of patients significantly declines [29]. However, many patients have an advanced cancer when they are diagnosed due to no obvious symptoms of early stage GC. Therefore, it is very necessary to elucidate the regulatory mechanisms of GC progression for seeking promising diagnostic markers and therapeutic targets. Here, we firstly reported that HOXA10-AS and HOXA10 were upregulated in GC, and HOXA10-AS enhanced malignant phenotypes of GC via upregulating HOXA10.

Increasing studies have validated vital roles of lncRNAs in the onset and development of GC in recent decades, showing the potential of lncRNAs to be applied or targeted in GC therapy [30, 31]. lncRNA ZEB1-AS1 was elevated in GC, and its overexpression indicated poor prognosis and facilitated metastasis [32, 33]. Mao and colleagues reported that lncRNA DANCR accelerated GC cell migration and invasion through inhibition of lncRNA LET [34]. Thus, revealing the biological activity of lncRNAs and identifying novel lncRNAs in cancers including GC are quite important.

HOXA10-AS plays an oncogenic role in several cancers. Sheng et al. found that HOXA10-AS could promote the proliferation and metastasis of lung adenocarcinoma cells via regulating the Wnt/*β*-catenin signaling [35]. However, the activity of HOXA10-AS in GC has not been reported. For the first time, we identified HOXA10-AS as a novel regulator in GC. Consistently, we found that HOXA10-AS acted as an oncogene to facilitate GC cell proliferation, migration, and invasion and reduce apoptosis, suggesting a crucial role of HOXA10-AS in GC tumorigenesis. High expression of HOXA10-AS was associated with poor survival of GC patients, suggesting potential clinical application of HOXA10-AS as a prognostic factor for GC.

RETRACTED

Several downstream targets of HOXA10-AS, including HOXA10 [16], NF-*κ*B target genes [15], and *β*-catenin [35], have been identified. Growing evidence has shown that HOXA10 functions as an oncogene. HOXA10 promoted invasion in pancreatic cancer [36], bladder cancer [37], and lung adenocarcinoma [38]. Importantly, emerging studies are uncovering the mystery of HOXA10 in stomach cancer. HOXA10 was upregulated in GC, and HOXA10 enhanced GC cell proliferation [39]. Moreover, HOXA10 served as a potential prognostic factor for GC [39, 40]. However, the role of HOXA10 in GC remains controversial. Sentani et al. found that overexpression of HOXA10 in GC with the intestinal mucin phenotype indicated good prognosis of patients [41]. In this study, our results showed that HOXA10 was upregulated by HOXA10-AS in GC and enhanced malignant phenotypes, supporting the oncogenic activity of HOXA10 in stomach cancer.

Taken together, we firstly demonstrated a novel role of the HOXA10-AS/HOXA10 axis in GC. In particular, HOXA10-AS enhanced malignant phenotypes of GC through upregulation of HOXA10. Our study not only sheds light on the role of HOXA10-AS in GC but also provides potential therapeutic targets. However, further investigations in animal models and patient samples are required to further evaluate the roles of the HOXA10-AS/HOXA10 axis in GC.

## Figures and Tables

**Figure 1:** HOXA10-AS was upregulated in GC. (a) TCGA database showed elevated HOXA10-AS expression in STAD. (b) qRT-PCR analysis of HOXA10-AS in NC and GC tissues (*n* = 70). (c) Overall survival of HOXA10-AS^high^ and HOXA10-AS^low^ patients was evaluated using the Kaplan-Meier curve (*p* < 0.01, HOXA10-AS^high^*n* = 35; HOXA10-AS^low^*n* = 35). (d) HOXA10-AS expression in HGC27, AGS, and GES-1 cells were examined using qRT-PCR (*n* = 3).

**Figure 2:** Knockdown of HOXA10-AS suppressed proliferation and enhanced apoptosis in GC cells. HGC27 and AGS cells were transfected with si-HOXA10-AS (#1, #2, or #3) or si-NC. (a) HOXA10-AS expression was assessed using qRT-PCR (*n* = 3). (b) Cell proliferation was determined by CCK-8 assay (*n* = 3). (c) EdU incorporation (red) in HGC27 and AGS cells (*n* = 3; scale bar, 100 *μ*m). The nucleus was stained with DAPI (blue). (d) Flow cytometry analysis of cell apoptosis (*n* = 3).

RETRACTED

**Figure 3:** Knockdown of HOXA10-AS suppressed migration and invasion in GC cells. (a) The wound healing assay was applied to examine cell migration (*n* = 3; scale bar, 100 *μ*m). Cell monolayers formed by HGC27 and AGS cells were scratched and incubated for healing. (b) The invasive capacity of HGC27 and AGS cells were evaluated using the transwell assay (*n* = 3; scale bar, 50 *μ*m). Crystal violet solution was used to stain invasive cells.

**Figure 4:** HOXA10-AS promoted HOXA10 expression in GC cells. (a) TCGA database showed elevated HOXA10 expression in STAD. (b) Correlation analysis of the expression of HOXA10-AS and HOXA10 in STAD using starBase v3.0. (c) qRT-PCR analysis of HOXA10 in NC and GC tissues (*n* = 70). (d) Spearman's correlation analysis of the expression of HOXA10-AS and HOXA10 in GC patients (*n* = 70, *p* < 0.001, *r* = 0.5540). (e) Western blot analysis of HOXA10 (*n* = 3).

**Figure 5:** HOXA10-AS accelerated malignant phenotypes of GC cells by promoting HOXA10 expression. HGC27 and AGS cells were transfected with empty vector (vector), HOXA10-AS-overexpressing vector (HOXA10-AS) or HOXA10-AS in combination with si-HOXA10. (a) HOXA10-AS expression was examined by qRT-PCR (*n* = 3). (b) Western blot analysis of HOXA10 (*n* = 3). (c) Cell proliferation was determined with CCK-8 assay (*n* = 3). (d) EdU incorporation (red) in HGC27 and AGS cells (*n* = 3; scale bar, 100 *μ*m). The nucleus was stained with DAPI (blue). (e) Flow cytometry analysis of cell apoptosis (*n* = 3). (f) The wound healing assay was applied to examine cell migration (*n* = 3; scale bar, 100 *μ*m). (g) The invasive capacity of HGC27 and AGS cells were examined using the transwell assay (*n* = 3; scale bar, 50 *μ*m).

**Table 1:** Correlation between HOXA10-AS expression and the clinical pathological features of gastric cancer patients.

Characteristic	All cases	HOXA10-AS expression		*p* value
		High (*n* = 35)	Low (*n* = 35)	
Age (years)				0.473
<60	33	15	18	
≥60	37	20	17	
Gender				0.629
Female	30	16	14	
Male	40	19	21	
Tumor size (cm)				0.151
<3	34	14	20	
≥3	36	21	15	
Lymph node metastasis				0.002^∗^
Yes	37	12	25	
No	33	23	10	
TNM				0.031^∗^
I+II	37	14	23	
III+IV	33	21	12	
Histological type				0.008^∗^
Well differentiated	37	13	24	
Poorly differentiated	33	22	11	

^∗^ *p* < 0.05.

## Data Availability

The data used to support the findings of this study are available from the corresponding author upon request.

RETRACTED

## Supplementary Materials

Supplementary Materials Supplementary Table 1: qRT-PCR primers in this study.
